This article has been retracted.

# Association study of inflammatory cytokine and chemokine expression in hand foot and mouth disease

**DOI:** 10.18632/oncotarget.18341

**Published:** 2017-06-02

**Authors:** Wenzhong Shang, Suying Qian, Lijuan Fang, Yong Han, Cuiping Zheng

**Affiliations:** ^1^ People’s Hospital of Fuyang District, Hangzhou, Zhejiang, P. R. China; ^2^ The Second Hospital of Ningbo, Ningbo, Zhejiang, P. R. China; ^3^ The Fourth Hospital of Xiaoshan District, Hangzhou, Zhejiang, P. R. China; ^4^ Key Laboratory of Tumor Molecular Diagnosis and Individualized Medicine of Zhejiang Province, Zhejiang Provincial People’s Hospital, Hangzhou, Zhejiang, P. R. China; ^5^ Dingli Hospital of Wenzhou Medical School, Wezhou Central Hospital, Zhejiang, P. R. China

**Keywords:** hand, foot and mouth disease, enterovirus 71, inflammatory cytokines, chemokines

## Abstract

**Objective:**

To determine the relationship of cytokine/chemokine expression with the clinical presentation of hand, foot and mouth disease (HFMD).

**Results:**

All cytokine/chemokine levels were higher in severe HFMD patients than in mild HFMD patients or controls (*P* < 0.01). RANTES, MCP-1, IL-4, IL-12 and IL-18 levels were higher in mild HFMD patients than in the controls (*P* < 0.05). In severe HFMD, all levels (except IL-8 and IL-4) were higher in patients with encephalitis plus pulmonary edema than in those with encephalitis alone (*P* < 0.05). All levels (except IL-8) were higher in EV71-positive patients than in EV71-negative patients (*P* < 0.05). In mild HFMD, all levels (except IL-8 and IL-4) were higher in EV71-positive patients than in EV71-negative patients (*P* < 0.05). In severe HFMD, only RANTES, IP-10 and IFN-γ levels were higher in EV71-positive patients than in EV71-negative patients (*P* < 0.05). In the EV71-negative group, all levels were higher in severe HFMD than in mild HFMD (*P* < 0.01). In the EV71-positive group, all levels (except IL-8) were higher in severe HFMD than in mild HFMD (*P* < 0.01).

**Materials and Methods:**

This study involved 28 mild HFMD patients, 44 severe HFMD patients and 26 healthy children. Venous blood was tested for cytokines (IL-4, IL-12, IL-18, TNF-α, IFN-γ) and chemokines (IL-8, RANTES, MCP-1, IP-10). Stool samples from the patients were tested for EV71 nucleic acid using reverse transcription polymerase chain reaction.

**Conclusions:**

Cytokines/chemokines participate in HFMD pathogenesis, and could have potential value in monitoring disease progression and predicting prognosis.

## INTRODUCTION

Hand, foot and mouth disease (HFMD) is a common acute infectious disease caused by a variety of human intestinal viruses. HFMD usually affects preschool children (age < 5 years) and has caused widespread epidemics in this population in recent years [1]. It is commonly caused by enterovirus 71 (EV71) and coxsackievirus A16 [2]. The severity of HFMD varies. Patients with mild HFMD present only mild fever and a self-limiting herpetic rash on the hands, feet and mouth. In patients with severe HFMD, however, the disease progresses rapidly, and may involve meningitis, brainstem encephalitis, pulmonary angioneurotic edema, pulmonary hemorrhage, myocarditis and even cardiopulmonary failure and death [3, 4].

The pathogenesis of severe HFMD caused by EV71 infection is not fully understood. Many studies have shown that cellular and humoral immune dysfunction in HFMD patients, in particular, the abnormal expression of inflammatory cytokines and chemokines and an imbalance in the expression of anti- and pro-inflammatory cytokines play an important role in the exacerbation of HFMD [5–10].

In this study, we determined the expression levels of inflammatory cytokines and chemokines in peripheral blood samples obtained from children with HFMD caused by EV71 infection. We analyzed the relationship of abnormal cytokine/chemokine expression levels with various clinical presentations of HFMD in order to clarify the mechanism underlying the exacerbation of HFMD. The potential clinical significance of the results is discussed.

## RESULTS

### Demographic data

Of the 72 samples (39 boys, 33 girls, average age 2.2 ± 0.7 years old, range from 1.2 to 4.1), 28 (17 boys, 11 girls, average age 2.3 ± 0.6 years old, range from 1.1 to 3.8) had mild HFMD and 44 (22 boys, 22 girls, average age 2.0 ± 0.9 years old, range from 1.0 to 4.3) had severe HFMD. The control group included 16 boys and 10 girls, with an average age of 2 ± 0.6 years old (range from 1.3 to 3.4 years old). No significant differences in age or sex were present between the mild HFMD, severe HFMD and control groups.

### Cytokine and chemokine expression

The plasma expression levels of all chemokines tested (IL-8, RANTES, MCP-1, IP-10; Figure 1A) and all cytokines tested (IL-4, IL-12, IL-18, TNF-α, IFN-γ; Figure 1B) were significantly higher in the severe HFMD group than in the mild HFMD and normal control groups (*P* < 0.01). The expression levels of the chemokines RANTES and MCP-1 (Figure 1A) and the cytokines IL-4, IL-12 and IL-18 (Figure 1B) were significantly higher in the mild HFMD group than in the normal control group (*P* < 0.05).

**Figure 1:** The expression of inflammatory **(A)** chemokines and **(B)** cytokines in children with severe and mild HFMD. *P < 0.05, **P < 0.01.

The children in the severe HFMD group were further divided into those with encephalitis (E group; *n* = 26; 14 boys, 12 girls) and those with both encephalitis and pulmonary edema (E + P group; *n* = 18; 8 boys, 10 girls). The plasma expression levels of all chemokines (except IL-8; Figure 2A) and cytokines (except IL-4; Figure 2B) were significantly higher in the E+P group than in the E group (*P <* 0.05).

**Figure 2:** The expression of inflammatory **(A)** chemokines and **(B)** cytokines in children with severe HFMD. E, encephalitis group; E+P, encephalitis with pulmonary edema group. *P < 0.05, **P < 0.01.

### EV71 nucleic acid detection in stool and its correlation with plasma cytokine/chemokine expression

We analyzed stool samples from the children with HFMD for the presence of EV71 nucleic acid by using RT-PCR assays. The plasma expression levels of all chemokines (except IL-8; Figure 3A) and cytokines (Figure 3B) tested were significantly higher in children whose stool samples tested positive for EV71 nucleic acid than in children whose stool samples were negative for EV71 nucleic acid (*P <* 0.05; Table 1). In the mild HFMD group, the plasma expression levels of all chemokines (except IL-8; Figure 4A) and cytokines (except IL-4; Figure 4B) were significantly higher in the EV71-positive patients than in the EV71-negative patients (*P <* 0.05). However, in the severe HFMD group, the expression levels of only RANTES, IP-10 and IFN-γ were significantly higher in the EV71-positive patients than in the EV71-negative patients (*P <* 0.05; Figure 4).

**Figure 3:** The expression of inflammatory **(A)** chemokines and **(B)** cytokines in HFMD patients whose stool samples tested positive or negative for EV71 nucleic acid. *P < 0.05, **P < 0.01.

**Table 1:** HFMD groups and EV71 status

Group	EV71-PCR (+)		EV71-PCR (−)	
	No. (M/F)	Average age (yr)	No. (M/F)	Average age (yr)
Mild	11 (7/4)	2.3 ± 0.8	17 (10/7)	2.2 ± 0.9
Severe (E)	17 (8/9)	1.9 ± 0.7	9 (6/3)	2.1 ± 0.6
Severe (E+P)	11 (6/5)	2.1 ± 0.8	7 (2/5)	2.2 ± 0.6

**Figure 4:** The expression of inflammatory **(A)** chemokines and **(B)** cytokines in the mild and severe HFMD groups according to EV71 status. *P < 0.05, **P < 0.01.

We regrouped the children with HFMD according to their EV71 status (positive vs. negative). Of the 72 study patients, 33 (18 boys, 15 girls) were EV71 negative, and 39 (21 boys, 18 girls) were EV71 positive. Of the 33 EV71-negative patients, 17 (10 boys, 7 girls) had mild HFMD and 16 (8 boys, 8 girls) had severe HFMD. Of the 39 EV71-positive patients, 11 (7 boys, 4 girls) had mild HFMD and 28 (14 boys, 14 girls) had severe HFMD.

In the EV71-negative group, the plasma expression levels of all cytokines and chemokines tested were significantly higher in children with severe HFMD than in children with mild HFMD (*P <* 0.01; Figure 5). In the EV71-positive group, the plasma expression levels of all cytokines and chemokines (except IL-8) were significantly higher in children with severe HFMD than in children with mild HFMD (*P <* 0.01; Figure 5).

**Figure 5:** The expression of inflammatory **(A)** chemokines and **(B)** cytokines in the EV71-positive and EV71-negative groups according to severity of HFMD. *P < 0.05, **P < 0.01.

## DISCUSSION

The immune system is a complex, sophisticated and coordinated network, whose dynamic equilibrium sustains health. Upon invasion by microorganisms, inflammatory mediators are generated in “signaling cascades” through a series of pathways and result in systemic inflammatory response syndrome. However, the excessive generation of inflammatory mediators can lead to tissue and organ damage; therefore, a variety of anti-inflammatory mediators are produced to inhibit excessive inflammatory responses and protect the body from immune damage [11]. Pro- and anti-inflammatory mediators coexist in the infection-induced immunological stress response, and the growth, decline and equilibrium of the two determine the evolution, development and prognosis of the infectious disease [12].

Children are a special group since their immune systems are not fully developed, which can be an important factor facilitating invasion by pathogenic microorganisms. Thus, children, especially preschoolers, are in a physiological immunocompromised state, and their specific and non-specific immune responses are poorer than those of adults. This may partly explain why preschoolers are susceptible to HFMD.

After EV71 infection, susceptible cells and non-specific immune cells are stimulated first to produce cytokines such as IFNs, TNF-α and IL-12. These cytokines play an important role in the early control of viral replication and infection. The virus further induces the production of chemokines, such as IL-8, MCP-1 and IP-10, which can contribute to the recruitment of non-specific immune cells, such as natural killer cells, monocytes and macrophages, to the infection site. Furthermore, the activation of these cells by cytokines leads to the secretion of inflammatory mediators and cytokines, interferes with viral replication and kills virus-infected host cells. These responses thus expand and enhance anti-infection immunity and accelerate recovery from HFMD, leading to a self-limiting disease [7, 10, 13–15]. The pathogenic mechanism that leads to the exacerbation of EV71 infection and to abnormal cytokine expression remains unknown.

In this study, we examined the relationship of plasma cytokine (IL-4, IL-12, IL-18, TNF-α, IFN-γ) and chemokine (IL-8, RANTES, MCP-1, IP-10) levels with disease severity (mild vs. severe groups), complications (E vs. E+P groups) and fecal EV71 status (EV71-positive vs. EV71-negative groups) in children with HFMD. Our results indicate that cytokines/chemokines participate in HFMD pathogenesis, and could be of potential value in monitoring disease progression and predicting prognosis.

Recent studies have shown that cytokines have inhibitory effects on the replication and infective ability of virus [16, 17], and that these cytokines are the major components of the early non-specific immune response to viral infections. In contrast, chemokines such as IL-8, RANTES, MCP-1 and IP-10 play important roles in the recruitment and activation of immune cells [18], thereby further enhancing anti-viral immunity. Overexpression or imbalance in the expression of these immune factors can aggravate the inflammatory response to infection, causing damage to infected tissues and leading to loss or disorders of organ function. Under these circumstances, the vulnerable immune system of children is unable to effectively eliminate the virus and control inflammation, which leads to further spread of the virus and eventually causes severe HFMD.

Lin et al. [6] confirmed the above mechanism by showing that the peripheral expression levels of IL-1β and several other inflammatory cytokines were significantly higher in the EV71-induced HFMD patients with both encephalitis and pulmonary edema than in those with only encephalitis, those with mild symptoms or normal controls. Wang et al. [7, 19] reported similar results; they found that the expression levels of inflammatory cytokines such as IFN-γ, MCP-1 and IP-10 in the peripheral blood and cerebrospinal fluid were significantly higher in patients with encephalitis and pulmonary edema than in patients with encephalitis or patients with mild disease.

Therefore, we believe that in the early stages of infection, the increase in the levels of various cytokines and chemokines may contribute to the early activation of specific and non-specific immunity. This maximizes the mobilization of various types of immune cells to participate in anti-EV71 infection immunity for the alleviation of or recovery from the disease. When the immune system cannot effectively clear the virus and control inflammation, the disease is exacerbated. Overexpression of inflammatory cytokines and chemokines in infected tissues can induce excessive immune responses and cause cytokine cascade reaction and cytokine storm through autocrine and paracrine mechanisms, resulting in severe local and systemic inflammation, and eventually tissue damage and organ dysfunction.

In conclusion, during the development and progression of HFMD, a variety of cytokines and chemokines are involved in the occurrence of inflammation. Some of these compounds clear the virus, while others exacerbate the disease. However, the immune pathogenesis of HFMD, its cytokine expression patterns and the changes in these patterns are not very clear at present. Further investigation into the roles of HFMD-related cytokines and chemokines in the pathogenesis of the disease is required to search for cytokine indices that can be used to monitor disease progression, determine prognosis and guide clinical diagnosis and treatment.

## MATERIALS AND METHODS

### Patient selection

This study involved 72 children with mild or severe HFMD who were treated at Hangzhou Sixth People’s Hospital between March 2011 and June 2012. All diagnoses were made using the Foot and Mouth Disease Treatment Guidelines (2010) issued by the Ministry of Health and the Expert Consensus on the Clinical Treatment of Severe Enterovirus 71 (EV71) Infection. Patients who received immunomodulators or had other viral or bacterial infections, or immune disorders were excluded. We also recruited 26 healthy children (control group) who had normal findings on physical examination from the same hospital. The collection of tissue specimens was approved and supervised by the research ethics committee of Hangzhou Sixth People’s Hospital. Written informed consents were obtained from all patients prior to operation.

### Sample collection

We collected venous blood samples (3 ml) from all children in the HFMD group and control group within 24 h of admission. The blood samples were collected in EDTA tubes and centrifuged (at 1300 g for 10 min) to obtain plasma samples, which were stored at −80°C until analysis. In addition, stool samples were collected from the children with HFMD and subjected to reverse transcription polymerase chain reaction (RT-PCR) assays for the detection of EV71 nucleic acid.

### Cytokine and chemokine detection

The plasma expression levels of the cytokines interleukin (IL)-4, IL-12, IL-18, tumor necrosis factor (TNF)-α and interferon (IFN)-γ and the chemokines IL-8, regulated on activation, normal T expressed and secreted (RANTES), monocyte chemotactic protein (MCP)-1 and IFN-γ–inducible protein (IP)-10 were determined using double-antibody sandwich enzyme-linked immunosorbent assay (R&D Systems, USA), according to the manufacturer’s instructions.

### Statistical analysis

Data were analyzed using SPSS 21.0 statistical software (IBM Inc. USA) and presented as mean ± standard deviation ($\bar{x}$± s). Multi-sample means were compared using unpaired *t*-test. Correlation was analyzed using Pearson correlation. Differences were considered statistically significant at *P <* 0.05.

## Abbreviations

EV71: enterovirus 71
HFMD: hand, foot and mouth disease
IFN: interferon
IL: interleukin
IP-10: IFN-γ–inducible protein-10
MCP-1: monocyte chemotactic protein-1
RANTES: regulated on activation, normal T expressed and secreted
RT-PCR: reverse transcription polymerase chain reaction
TNF: tumor necrosis factor
